The article "5G Network Slicing: Methods to Support Blockchain and Reinforcement Learning" was published in 2022. Journal: Comput Intell Neurosci.

# 5G Network Slicing: Methods to Support Blockchain and Reinforcement Learning

**DOI:** 10.1155/2022/1164273

**Published:** 2022-03-24

**Authors:** Juan Hu, Jianwei Wu

**Affiliations:** ^1^School of Intelligent Engineering, Zhengzhou University of Aeronautics, Zhengzhou 450046, China; ^2^The 27th Research Institute of China Electronics Technology Group Corporation, Weishi 450047, China

## Abstract

With the advent of the 5G era, due to the limited network resources and methods before, it cannot be guaranteed that all services can be carried out. In the 5G era, network services are not limited to mobile phones and computers but support the normal operation of equipment in all walks of life. There are more and more scenarios and more and more complex scenarios, and more convenient and fast methods are needed to assist network services. In order to better perform network offloading of the business, make the business more refined, and assist the better development of 5G network technology, this article proposes 5G network slicing: methods to support blockchain and reinforcement learning, aiming to improve the efficiency of network services. The research results of the article show the following: (1) In the model testing stage, the research results on the variation of the delay with the number of slices show that the delay increases with the increase of the number of slices, but the blockchain + reinforcement learning method has the lowest delay. The minimum delay can be maintained. When the number of slices is 3, the delay is 155 ms. (2) The comparison of the latency of different types of slices shows that the latency of 5G network slicing is lower than that of 4G, 3G, and 2G network slicing, and the minimum latency of 5G network slicing using blockchain and reinforcement learning is only 15 ms. (3) In the detection of system reliability, reliability decreases as the number of users increases because reliability is related to time delay. The greater the transmission delay, the lower the reliability. The reliability of supporting blockchain + reinforcement learning method is the highest, with a reliability of 0.95. (4) Through the resource utilization experiment of different slices, it can be known that the method of blockchain + reinforcement learning has the highest resource utilization. The resource utilization rate of the four slices under the blockchain + reinforcement learning method is all above 0.8 and the highest is 1. (5) Through the simulation test of the experiment, the results show that the average receiving throughput of video stream 1 is higher than that of video stream 2, IOT devices and mobile devices, and the average cumulative receiving throughput under the blockchain + reinforcement learning method. The highest is 1450 kbps. The average QOE of video stream 1 is higher than that of video stream 2, IOT devices and mobile devices, and the average QOE is the highest under the blockchain + reinforcement learning method, reaching 0.83.

## 1. Introduction

Relieving users' network congestion, reducing network latency, and offloading the network are the top priorities for 5G networks. As a core technology, the 5G network slicing technology can effectively solve the challenges of business creation and exclusive network access for different users, as well as the coexistence of multiple application scenarios. The 5G network is expected to meet the different needs of users [1]. 5G network slicing may be a natural solution [2]. A wide range of services required for vertical specific use cases can be accommodated simultaneously on the public network infrastructure. 5G mobile networks are expected to meet flexible demands [3]. Therefore, network resources can be dynamically allocated according to demand. Network slicing technology is the core part of 5G network [4]. The definition of 5G network slicing creates a broad field for communication service innovation [5]. The vertical market targeted by 5G networks supports multiple network slices on general and programmable infrastructure [6]. The meaning of network slicing is to divide the physical network into two virtual networks so that they can be flexibly applied to different network scenarios. The future 5G network will also change the mobile network ecosystem [7]. The 5G mobile network is expected to meet the diversified needs of a variety of commercial services [8]. 5G mobile networks must support a large number of different service types [9]. Network slicing allows programmable network instances to be provided to meet the different needs of users. Blockchain can establish a secure and decentralized resource sharing environment [10]. Blockchain is a distributed open ledger [11] and is used to record transactions between multiple computers. Reinforcement learning algorithms can effectively solve large state spaces [12]. Reinforcement learning is mainly used to solve simple learning tasks [13]. 5G networks are designed to support many vertical industries with different performance requirements [14]. Network slicing is considered an important factor in enhancing the network and has the necessary flexibility to achieve this goal. Network slicing is considered one of the key technologies of 5G network [15]. You can create virtual networks and provide customized services on demand.

## 2. Overview of Related Theories

### 2.1. 5G Network Slicing

#### 2.1.1. Network Slicing

Network slicing refers to the implementation of offload management of the network when the network is congested and complicated [16]. When facing the different needs of different users, the network is divided into many pieces to meet customer needs. Moreover, it provides targeted services and assistance.

#### 2.1.2. Network Slice Classification

The ultimate goal of 5G network slicing is to organically combine multiple network resource systems to form a complete network that can serve different types of users. Network slices can be divided into independent slices and shared slices as shown in Table 1:

#### 2.1.3. 5G Network Application Scenarios

The application scenarios of 5G networks are divided into three categories: mobile broadband, massive Internet of Things, and mission-critical Internet of Things [17]. The details are shown in Table 2:

### 2.2. Blockchain

#### 2.2.1. Definition of Blockchain

The blockchain consists of a shared, fault-tolerant distributed database, and a multi-node network [18].

#### 2.2.2. Blockchain Structure

The block chain is composed of a block header and a block body, which forms into a chain structure through the hash of the parent block [19]. The structure is shown in Figure 1:

The structure contains the parent block hash, timestamp, random number, difficulty, and the Merkle root [20]. Its functions are shown in Table 3:

#### 2.2.3. Blockchain Properties

Blockchain technology has three attributes of distribution, security, and robustness [21], as shown in Table 4:

### 2.3. Reinforcement Learning

#### 2.3.1. Definition of Reinforcement Learning

Reinforcement learning is one of the methods of machine learning. It is mainly to solve the method of how the agent takes different actions in the environment in order to maximize the accumulated rewards obtained.

#### 2.3.2. Reinforcement Learning Process

In the process of reinforcement learning, the agent needs to make decisions on the information in the environment [22]. At the same time, the environment will also reward the agent for the corresponding behavior, and the agent will enter a new state after the behavior. The process is shown in Figure 2:

### 2.4. Model Design

The 5G network slicing architecture is composed of network slicing demander, slice management (business design, instance orchestration, operation management), slice selection function, and virtualization management orchestration.

The process of the 5G network slicing model is as follows: network services enter the slice manager through the network slice demander, and the slice manager includes business design, instance arrangement, and operation management. After the slice manager enters the slice selection function, it is divided into shared slice function and independent slice special function, and it can also enter the virtualization management orchestration as shown in Figure 3:

## 3. Formula

### 3.1. Blockchain

#### 3.1.1. Scalability within Shards

In the process of verifying the block consensus, the scalability within the shard [23]is as follows:

(1) $$\begin{array}{c} \Phi \left(B_{F},T_{F}\right)=\frac{\left|\left(B_{F}-B_{H}\right)/b_{F}\right|}{T_{F}}. \end{array}$$

Among them, *b*_*I*_ is the average transaction size, *B*_*Ih*_ is the block header size, and *K* is the number of shards.

#### 3.1.2. Scalability of Directory Fragmentation

Assuming that the average transaction size is *b*_*F*_, the block header size is *B*_*H*_, and the scalability of the directory fragmentation is as follows:

(2) $$\begin{array}{c} \Phi \left(B_{I},T_{II}\right)=\sum_{i=1}^{K}\frac{\left|\left(B_{I}-B_{Ih}\right)/b_{I}\right|}{T_{II_{i}}}. \end{array}$$

#### 3.1.3. Scalability of Sharded Blockchain

The scalability of the entire sharded blockchain is composed of the internal scalability of the shards and the scalability of the catalog shards [24]. Assuming that the block packing time within the fragment and the directory fragment is the same as *T*_*I*_′ and the block header size is the same as *B*_*H*_′, the formula is as follows:

(3) $$\begin{array}{c} \Phi \left(B,T\right)=\Phi \left(B_{I},T_{II}\right)+\Phi \left(B_{F},T_{F}\right)\\ \Phi \left(B,T\right)=\sum_{i=1}^{K}\frac{\left|\left(B_{I}-B_{Ih}\right)/b_{I}\right|}{T_{II_{i}}}+\frac{\left|\left(B_{F}-B_{h}\right)/b_{F}\right|}{T_{F}}\\ \Phi \left(B,T\right)=\frac{\left|k\left(B_{I}-B_{H}^{\prime }\right)/b_{I}+\left(B_{F}-B_{h}\right)/b_{F}\right|}{T_{I}^{\prime }}. \end{array}$$

### 3.2. Reinforcement Learning Methods

#### 3.2.1. Value Function Method

The value function method is to give an estimate of the value for different states. 0 is the given value, and *V*^*π*^(*s*) starts from state *V*^*π*^(*s*). The formula is as follows:

(4) $$\begin{array}{c} V^{\pi }\left(s\right)=E_{\pi }\left[R|s,\pi \right],\\ V^{\pi }\left(s\right)=E_{\pi }\left[R_{0}+\gamma R_{1}+\gamma^{2}R_{2}+\cdots +\gamma^{t}R_{t}+\cdots |s=S_{t}\right]. \end{array}$$

The optimal strategy *π*^*∗*^ has a corresponding state-value function *V*^*∗*^(*s*), which is expressed as follows:

(5) $$\begin{array}{c} V^{*}\left(s\right)=\max_{\pi }V^{\pi }\left(s\right)\forall s\in S. \end{array}$$

In the RL setting, it is difficult to obtain the state transition function *P*. So, a state-action value function is constructed.

(6) $$\begin{array}{c} Q_{\pi }\left(s,a\right)=E\left[R|s,a,\pi \right],\\ Q^{\pi }\left(s,a\right)=E\left[R_{0}+\gamma R_{1}+\gamma^{2}R_{2}+\cdots +\gamma^{t}R_{t}+\cdots |s=S_{t},a=A_{t}\right]. \end{array}$$

Given *Q*^*π*^(*s*, *a*), in each state, the optimal strategy argmax_*a*_*Q*^*π*^(*s*, *a*) can be adopted. Under this strategy, *V*^*π*^(*s*) can be defined by maximizing *Q*^*π*^(*s*, *a*)as follows:

(7) $$\begin{array}{c} V^{\pi }\left(s\right)=\max_{a}Q^{\pi }\left(s,a\right). \end{array}$$

At present, mature deep learning methods such as SARSA and offline *Q* learning can all be used to solve the value function.

SARSA:

(8) $$\begin{array}{c} Q\left(S_{t},A_{t}\right)\leftarrow Q\left(S_{t},A_{t}\right)+\alpha \left[R_{t+1}+\gamma \max_{a}Q\left(S_{t+1},a\right)-Q\left(S_{t},A_{t}\right)\right]. \end{array}$$

Offline *Q* learning:

(9) $$\begin{array}{c} Q\left(S_{t},A_{t}\right)\leftarrow Q\left(S_{t},A_{t}\right)+\alpha \left[R_{t+1}+\gamma Q\left(S_{t+1},A_{t+1}\right)-Q\left(S_{t},A_{t}\right)\right]. \end{array}$$

#### 3.2.2. Strategy Method

The strategy method is to directly output the action by searching for the optimal strategy *π*^*∗*^. The objective function *J*(*θ*) is defined as the cumulative expected reward.

(10) $$\begin{array}{c} J\left(\theta \right)=E\left[\sum_{t⟶0}^{\infty }\gamma^{t}r_{t}|\pi \right]=\int_{s}d^{\pi }\left(S\right)\int_{A}\pi \left(a|s,\theta \right)R\left(s,a\right)\text{d}s\text{d}a. \end{array}$$

The policy parameter ∇_*θ*_*J*(*θ*) is estimated in the discounted cumulative expected reward gradient *θ* and obtained based on a certain learning rate (*α*_*l*_). The formula of the strategy gradient method is as follows:

(11) $$\begin{array}{c} \theta_{l+1}=\theta_{l}+\alpha_{t}\nabla_{\theta }J\left(\theta \right){|}_{\theta -\theta_{l}}. \end{array}$$

#### 3.2.3. MDP

MDP mainly solves the problem of learning-related experiences in the interaction between the agent and the environment to achieve the goal [25]. Assuming that the state space is *S*, it is defined as follows:

(12) $$\begin{array}{c} S=\left\{\left(h,x,d,\varphi \right)|\forall h\in H,x\in X,d\in D,\varphi \in \psi \right\}. \end{array}$$

Among them, *h* represents the state of all wireless channels in the 5G network slice, *H* represents the channel state space, and *H* is represented as follows:

(13) $$\begin{array}{c} H=\left\{\left(h_{1},h_{2},\ldots ,h_{m}\right)|\forall m\in M,h_{m}\in H_{m}\right\}. \end{array}$$

Among them, *h*_*m*_ represents the channel state and *H*_*m*_ represents the channel state space.

*x* means connection status, *X* means connection status space. *X* is defined as follows:

(14) $$\begin{array}{c} X=\left\{\left(x_{1},x_{2},\ldots ,x_{\left|M\right|}\right)|\forall m\in M,x_{m}\in X_{m}\right\}. \end{array}$$

*d* represents the state of all data transmission rates in the slice, and *D* represents the data transmission rate state space. *D* is defined as follows:

(15) $$\begin{array}{c} D=\left\{\left(d_{1},d_{2},\ldots ,d_{\left|U\right|}\right)|\forall u\in U,d\in \left[d_{\min},d_{\max}\right]\right\}. \end{array}$$

*φ* represents the topological state of the physical network, and *ψ* represents the topological state space in the physical network. *ψ* is defined as follows:

(16) $$\begin{array}{c} \psi =\left\{\left(\varphi_{1},\varphi_{2},\ldots ,\varphi_{\left|N\right|}\right)|\forall \varphi \in \psi ,\varphi \in \left\{0,1\right\}\right\}. \end{array}$$

*A*_*r*_ means that the action space is allocated for unlimited resources, which is defined as follows:

(17) $$\begin{array}{c} A_{r}=\left\{\left(a_{r,1},a_{r,2},\ldots ,a_{r,\left|U\right|}\right)|\forall u\in U,a_{r,u}\in A_{r,u}\right\}. \end{array}$$

Among them, *a*_*r*,*u*_ is the 5G network radio resource allocation action, and *A*_*r*,*u*_ is its corresponding network action space, expressed as follows:

(18) $$\begin{array}{c} A_{r,u}=\left\{v_{u,m}^{\prime }|m\in M,v_{u,m}^{\prime }\in \left[0,v_{m}^{\prime }\right]\right\}. \end{array}$$

Among them, *v*_*u*,*m*_′ represents occupied wireless resources.

### 3.3. Model Building

Suppose the weighted undirected graph of the physical network is *C*=(*A*_*i*_, *S*_*i*_), where the set of network nodes is denoted as *A*_*i*_={*a*_1_, *a*_2_,…, *a*_*n*_}, the calculation level of *A*_*i*_ is denoted as *S*_*i*_={*s*_1_, *s*_2_,…, *s*_*n*_}, and the link set composed of nodes is denoted as *L*_*n*_={*l*_1_, *l*_2_,…, *l*_*n*_}.

The first dynamic dispatch queue state transition function is as follows:

(19) $$\begin{array}{c} Z\left(X\right)=\gamma_{i}+\left(A_{i}S_{i}-L_{n}\right)d_{i}. \end{array}$$

The second dynamic scheduling queue state transition function is as follows:

(20) $$\begin{array}{c} Z\left(Y\right)=\frac{\gamma_{i}+A_{i}L_{n}d_{i}}{Z\left(X\right)}. \end{array}$$

Combining the above analysis, the 5G network slicing model, the formula is expressed as below:

(21) $$\begin{array}{c} F\left(x\right)=\frac{Z\left(X\right)+Z\left(Y\right)}{d_{i}}\gamma_{i}. \end{array}$$

## 4. Experiment

### 4.1. Model Test

#### 4.1.1. Variation of Time Delay with the Number of Slices

This article mainly studies 5G network slicing methods to support blockchain and reinforcement learning. First, we will test the model and compare the blockchain + reinforcement learning method with the blockchain, reinforcement learning, and unused methods. The results are shown in Figure 4.

The comparison results show that the delay increases with the increase of the number of slices, but the blockchain + reinforcement learning method has the lowest delay and can maintain the minimum delay. When the number of slices is 3, the delay is 155 ms. The overall delay of the blockchain is lower than the delay of reinforcement learning because the blockchain will give priority to nodes with rich resources and strong data processing capabilities when selecting nodes and link mappings, so the delay is lower.

#### 4.1.2. Delay Comparison of Different Slice Types

Under different slice types, set the number of users to 30 and compare the delays generated by several methods. We compare 5G network slicing, 4G network slicing, 3G network slicing, and 2G network slicing in blockchain + reinforcement learning, blockchain, reinforcement learning, and unused methods. The results are shown in Figure 5.

Through the comparison results, it can be seen that the latency of 5G network slicing is lower than that of 4G, 3G, and 2G. 5G network slicing has the lowest latency of only 15 ms in the method of blockchain and reinforcement learning. This is because the greater the number of VNFs, the more nodes that the slice will pass through to process the same data packet, the longer the link that passes, and the greater the delay.

#### 4.1.3. System Reliability

System reliability is an indispensable step before the experiment. We will compare the system reliability of different methods (blockchain + reinforcement learning, blockchain, reinforcement learning) under different numbers of users. The comparison result is shown in Figure 6:

It can be seen from the graph that the reliability decreases with the increase of the number of users because reliability is related to delay. The greater the transmission delay, the lower the reliability. The reliability of the supporting blockchain + reinforcement learning method is the highest, with a reliability of 0.95. This means that 5G network slicing that supports blockchain + reinforcement learning methods can provide services for more businesses.

### 4.2. Resource Utilization of Different Slices

This article studies the methods that support blockchain and reinforcement learning. We will study the resource utilization of blockchain and reinforcement learning for different slices. Set up 4 slices and perform three tests on each slice, namely, blockchain + reinforcement learning, blockchain and reinforcement learning, and finally compare their resource utilization experiment results as shown in Figure 7:

According to the experimental results, it can be concluded that the method of blockchain + reinforcement learning has the highest resource utilization rate. The resource utilization rate of the four slices under the blockchain + reinforcement learning method is all above 0.8, and the highest is 1. It shows that the block chain + reinforcement learning method has the best resource utilization for the block.

### 4.3. Simulation Test

According to the 5G network proposed in this article: Support blockchain and reinforcement learning methods to design a simulation test. Excluding other factors, the experimental subjects are video stream 1, video stream 2, IOT devices, and mobile devices.

#### 4.3.1. Average Cumulative Receiving Throughput

The experiment will compare 4 types of equipment using three methods: blockchain + reinforcement learning, blockchain, and reinforcement learning. By comparing the average cumulative received throughput (kpbs), which method is better is decided. Throughput refers to the number of requests processed by the system in a unit of time. The results are shown in Table 5.

The result is plotted as a histogram, and the result is shown in Figure 8.

According to the experimental results, the average receiving throughput of video stream 1 is higher than that of video stream 2, IOT devices, and mobile devices, and the average cumulative receiving throughput is the highest under the blockchain + reinforcement learning method, reaching 1450 kbps.

#### 4.3.2. Average QOE

Under three different methods, compare the average QOE of different devices to prove which method is more suitable for 5G network slicing. QOE refers to the user's comprehensive experience of the quality and performance of the network system. The results are shown in Table 6:

The result is plotted as a histogram, and the result is shown in Figure 9.

According to the experimental results, the average QOE of video stream 1 is higher than that of video stream 2, IOT devices, and mobile devices, and the average QOE is the highest under the blockchain + reinforcement learning method, reaching 0.83.

## 5. Conclusion

With the advent of the 5G era, current technologies can no longer meet the needs of users. Network congestion and slow network speeds are major problems currently facing. In order for users to use network services more smoothly, network services are more convenient. This article designs 5G network slicing: a method model supporting blockchain and reinforcement learning. This model will perform better distribution management of the network, increase the transmission rate of users in the business, and reduce the transmission delay.

The research results of the article are given below:

1. In the model testing stage, the results of the study on the variation of the delay with the number of slices show that the delay increases with the increase of the number of slices, but the blockchain + reinforcement learning method has the lowest delay and can maintain the minimum delay When the number of slices is 3, the delay is 155 ms.
2. The comparison of the delay of different slice types shows that the delay of 5G network slicing is lower than that of 4G, 3G, and 2G. 5G network slicing has the lowest delay in the method of blockchain and reinforcement learning, only 15 ms.
3. In the detection of system reliability, reliability decreases as the number of users increases. This is because reliability is related to delay. The greater the transmission delay, the lower the reliability. Supporting blockchain + reinforcement learning method has the highest reliability.
4. In the resource utilization experiment of different slices, it can be known that the method of blockchain + reinforcement learning has the highest resource utilization. The resource utilization rate of the four slices under the blockchain + reinforcement learning method is all above 0.8 and the highest is 1.
5. Through the simulation test of the experiment, the results show that the average receiving throughput of video stream 1 is higher than that of video stream 2, IOT devices, and mobile devices, and the average cumulative receiving throughput under the blockchain + reinforcement learning method The volume is the highest, reaching 1450 kbps. The average QOE of video stream 1 is higher than that of video stream 2, IOT devices, and mobile devices, and the average QOE is the highest under the blockchain + reinforcement learning method, reaching 0.83.

Although the results of this experiment are obvious, it has certain limitations and is limited to the use of 5G network slicing. A lot of research is needed in the future to enhance its universality and apply it to more scenarios. In future research, the methods for supporting blockchain and reinforcement learning proposed in this article can be improved, so that blockchain and reinforcement learning methods can be realized in the network service requirements with more goals.

## Figures and Tables

**Figure 1:** Blockchain structure.

**Figure 2:** Reinforcement learning process.

**Figure 3:** Model design.

**Figure 4:** Time delay changes with the number of slices.

**Figure 5:** Delay comparison of different slice types.

**Figure 6:** System reliability.

**Figure 7:** Resource utilization of different slices.

**Figure 8:** Average cumulative receiving throughput.

**Figure 9:** Average QOE.

**Table 1:** Network slice classification.

Independent slice	A slice with a logically independent and complete network function. The slice includes a user data plane, a network control plane, and various user business function films, which can provide a logically independent end-to-end private network service for a specific user group. If necessary, only part of the services of specific functions can be provided.
Shared slice	A shared slice is a specific network slice whose network resources can be used by different independent slices. The slice can provide end-to-end services, and when necessary, it can also only provide partial sharing functions.

**Table 2:** 5G network application scenarios.

5G application scenarios	Application examples	Need
Mobile broadband	4K/8K Ultra HD video, holographic technology, augmented reality/virtual reality	High capacity, video storage
Mass Internet of Things	Massive sensors (deployed in measurement, construction, agriculture, logistics, smart cities, homes, etc.)	Large-scale connection (200,000/km^2^), mostly stationary
Mission Critical Internet of Things	Autonomous driving, automated factories, smart grids, etc.	Low latency, high reliability

**Table 3:** Blockchain structure function.

Parent block hash	Has the hash value of the previous block
Timestamp	Used to record the time when the current block was generated
Random number and difficulty	Used to calculate proof of work
Version number	Record the version of the current block, so that you can view and update the version at any time
Merkle root value of the entire block	It is the root value of the Merkle tree, which stores the hash value of all transactions in the entire block

**Table 4:** Blockchain attributes.

Distributed	The blockchain connects the participating nodes through a peer-to-peer network to realize resource sharing and task allocation between peer nodes. Each network node does not need to rely on the central node and can directly share and exchange information. Each peer node can not only be an acquirer of services, resources, and information but can also be a provider thereof, which reduces the complexity of networking while improving the fault tolerance of the network.
Safety	Blockchain can use encryption technology to asymmetrically encrypt the transmitted data information. The task request for writing data in the blockchain needs to be accompanied by the private key signature of the task initiator. The changed signature is broadcasted together with the task request among participating nodes in the network. Each node can verify its identity, so the task request is not allowed for forgery and tampering. At the same time, the blockchain data structure in the blockchain further ensures that the content in the block cannot be tampered with at will. Even if some nodes in the chain are maliciously forged, tampered with, or destroyed. It will not affect the normal operation of the entire blockchain.
Robustness	The consensus mechanism determines the degree of agreement between the voting weight and computing power between subjects. The entire blockchain system uses a special incentive mechanism to attract more miners to participate in the process of generating and verifying data blocks, perform mathematical calculations in a distributed system structure, use consensus algorithms to select a node, and then create a new one. The effective block of is added to the entire blockchain, and the entire process does not rely on a third-party trusted institution.

**Table 5:** Average cumulative receiving throughput.

Equipment	Blockchain + reinforcement learning	Blockchain	Reinforcement learning
Video stream 1	1450	1400	1150
Video stream 2	1350	1320	1160
IOT equipment	700	650	480
Mobile devices	270	260	100

**Table 6:** Average QOE.

Equipment	Blockchain + reinforcement learning	Blockchain	Reinforcement learning
Video stream 1	0.83	0.75	0.68
Video stream 2	0.79	0.73	0.62
IOT equipment	0.7	0.64	0.47
Mobile devices	0.64	0.56	0.4

## Data Availability

The experimental data used to support the findings of this study are available from the corresponding author upon request.

## References

[1] Zhang H., Liu N., Chu X., Long K., Aghvami A.-H., Leung V. C. M. (2017). Network slicing based 5G and future mobile networks: Mobility, resource management, and challenges. *IEEE Communications Magazine*.

[2] Ordonez-Lucena J., Ameigeiras P., Lopez D., Ramos-Munoz J. J., Lorca J., Folgueira J. (2017). Network slicing for 5G with SDN/NFV: Concepts, architectures, and challenges. *IEEE Communications Magazine*.

[3] Jiang M., Condoluci M., Mahmoodi T. Network slicing management & prioritization in 5G mobile systems.

[4] Luo M., Wu J., Li X. (2020). Cross-domain certificateless authenticated group key agreement protocol for 5G network slicings. *Telecommunication Systems: Modelling, Analysis, Design and Management*.

[5] Kourtis M. A., Sarlas T., Xilouris G. (2021). Conceptual evaluation of a 5G network slicing technique for emergency communications and preliminary estimate of energy trade-off. *Energies*.

[6] Campolo C., Molinaro A., Iera A. (2018). 5G network slicing for vehicle-to-everything services. *IEEE Wireless Communications*.

[7] Bega D., Gramaglia M., Banchs A., Sciancalepore V., Samdanis K., Costa-Perez X. Optimising 5G infrastructure markets: the business of network slicing.

[8] Jiang M., Condoluci M., Mahmoodi T. Network slicing in 5G: An auction-based model.

[9] Pries R., Morper H. J., Galambosi N., Jarschel M. Network as a service-a demo on 5G network slicing.

[10] Dai Y., Xu D., Maharjan S., Chen Z., He Q., Zhang Y. (2019). Blockchain and deep reinforcement learning empowered intelligent 5G beyond. *IEEE Network*.

[11] Ahamed N. N., Karthikeyan P. (2020). A reinforcement learning integrated in heuristic search method for self-driving vehicle using blockchain in supply chain management. *International Journal of Intelligent Networks*.

[12] Nguyen D. C., Pathirana P. N., Ding M., Seneviratne A. (2020). Privacy-preserved task offloading in mobile blockchain with deep reinforcement learning. *IEEE Transactions on Network and Service Management*.

[13] Long-Ji L. (1992). Self-improving reactive agents based on reinforcement learning, planning and teaching. *Machine Learning*.

[14] Kaloxylos A. (2018). A survey and an analysis of network slicing in 5G networks. *IEEE Communications Standards Magazine*.

[15] Jia Q., Xie R., Huang T., Liu J., Liu Y. (2017). Efficient caching resource allocation for network slicing in 5G core network. *IET Communications*.

[16] Stone P., Sutton R. S., Kuhlmann G. (2005). Reinforcement learning for RoboCup soccer keepaway. *Adaptive Behavior*.

[17] Chen G., Qi J., Tang C., Wang Y., Wu Y., Shi X. (2020). Analysis and research of key genes in gene expression network based on complex network. *Complexity*.

[18] Ning X., Gong K., Li W., Zhang L. (2021). JWSAA: Joint weak saliency and attention aware for person re-identification. *Neurocomputing*.

[19] Theodorou A., Buchli J., Sch A. L. S. (2010). A generalized path integral control approach to reinforcement learning. *Journal of Machine Learning Research*.

[20] Yuan Y., Wang F. Y. (2016). Blockchain: The state of the art and future trends. *Acta Automatica Sinica*.

[21] Sun L., Yu Q., Peng D., Subramani S., Wang X. (2021). FogMed: a fog-based framework for disease prognosis based medical sensor data streams. *Computers, Materials & Continua*.

[22] Verbert K., Sharples M., Klobuar T. The blockchain and kudos: A distributed system for educational record, reputation and reward.

[23] Abidi M. H., Alkhalefah H., Moiduddin K. (2021). Optimal 5G network slicing using machine learning and deep learning concepts. *Computer Standards & Interfaces*.

[24] Tobar C. H., Ordonez A., Rendon O. (2020). Scalability and performance analysis in 5G core network slicing. *IEEE Access*.

[25] Tang L., Zhou Y., Yang Y. (2019). Virtual network function dynamic deployment algorithm based on prediction for 5G network slicing. *Journal of Electronics and Information Technology*.

